RETRACTED

# Identification of Hub Genes for Early Diagnosis and Predicting Prognosis in Colon Adenocarcinoma

**DOI:** 10.1155/2022/1893351

**Published:** 2022-06-21

**Authors:** Shuo Xu, Dingsheng Liu, Mingming Cui, Yao Zhang, Yu Zhang, Shiqi Guo, Hong Zhang

**Affiliations:** Department of General Surgery, Shengjing Hospital of China Medical University, 36 Sanhao Street, Heping District, Shenyang 110004, China

## Abstract

Colon adenocarcinoma (COAD) is among the most common digestive system malignancies worldwide, and its pathogenesis and gene signatures remain unclear. This study explored the genetic characteristics and molecular mechanisms underlying colon cancer development. Three gene expression data sets were obtained from the Gene Expression Omnibus (GEO) database. GEO2R was used to determine differentially expressed genes (DEGs) between COAD and normal tissues. Then, the intersection of the data sets was obtained. Metascape was used to perform the functional enrichment analyses. Next, STRING was used to build protein-protein interaction (PPI) networks. Hub genes were identified and analysed using Cytoscape. Next, survival analysis and expression analysis of the hub genes were performed. ROC curve analysis was performed for further test of the diagnostic efficacy. Finally, alterations in the hub genes were predicted and analysed by cBioPortal. Altogether, 436 DEGs were detected. The DEGs were mainly enriched in cell cycle phase transition, nuclear division, meiotic nuclear division, and cytokinesis. Based on PPI networks, 20 hub genes were selected. Among them, 6 hub genes (*CCNB1*, *CCNA2*, *AURKA*, *NCAPG*, *DLGAP5*, and *CENPE*) showed significant prognostic value in colon cancer (*P* < 0.05), while 5 hub genes (*CDK1*, *CCNB1*, *CCNA2*, *MAD2L1*, and *DLGAP5*) were associated with early colon cancer diagnosis and ROC curve analysis showed good diagnostic accuracy. In conclusion, integrated bioinformatics analysis was used to identify hub genes that reveal the potential mechanism of carcinogenesis and progression of colon cancer. The hub genes might be novel biomarkers for early diagnosis, treatment, and prognosis of colon cancer.

## 1. Introduction

Colon adenocarcinoma (COAD) is among the most common digestive system malignancies worldwide. There were 1,096,601 new colon cancer cases and 551,269 deaths worldwide in 2018 [1]. In the last decade, both the incidence and mortality of colon cancer increased in rapidly transitioning countries including the Baltic countries, Russia, China, and Brazil [2]. As previously reported, the 5-year survival rate was more than 90% for patients diagnosed with stage I, but only 12% for patients diagnosed with stage IV [3]. Thus, early diagnosis and surgical resection of colon cancer will greatly improve disease prognosis. The current early screening tests included noninvasive tests of stool and blood-based tests, radiologic tests, and invasive test like colonoscopy. However, the participation and adherence rates of screening were low, mainly due to the unreliable accuracy of noninvasive tests and low acceptance of the invasive tests as well as the expensive cost [4]. Computed tomographic colonography (CTC) with bowel preparation was reported to have a diagnostic sensitivity of 68.5% and specificity of 88.8% for adenoma ≥ 6 mm, while overall sensitivity (55.3%) and specificity (34.1%) were much lower for adenomas of all sizes [5]. Another study reported that the sensitivity of faecal immunochemical test (FIT) in detecting adenoma, advanced neoplasm, and cancer was 9.5%, 35.1%, and 25.0%, respectively, which showed a low diagnostic accuracy [6]. As a result, only 39% of tumours were diagnosed at an early stage, and the colon cancer remained a serious health burden worldwide [7]. Thus, it is essential to uncover the molecular mechanism and to explore novel biomarkers for early colon cancer diagnosis.

RETRACTED

At present, molecular biomarkers are mainly divided into three categories [8]: prognostic biomarkers such as tumour suppressor p53, vascular endothelial growth factor (*VEGF*), and epidermal growth factor receptor (*EGFR*); diagnostic biomarkers such as telomerase and pyruvate kinase M2 (*PKM2*); and predictive biomarkers such as *KRAS* and *B-Raf V600E*. Currently, some molecular markers have been applied in clinical practice. A study confirmed prostaglandin E receptor 4 (PTGER4)/short stature homeobox 2 (SHOX2) DNA methylation as a biomarker for early detection of lung cancer [9]. The panel of trefoil factor (TFF) 1, TFF2, and TFF3 may be potential biomarkers for early screening of breast cancer [10]. However, the accuracy and reliability of many markers were not satisfactory [8, 11]. Therefore, it is urgent to explore a single or a series of accurate and effective markers for early diagnosis and better individualized treatment of colon cancer [12]. RNA sequencing and gene expression microarrays were widely applied in cancer studies. Bioinformatics analysis of these data can be used to identify significant biomarkers which may improve cancer early diagnosis, predict prognosis, and inform therapeutic responses [13, 14]. Although there were some previous studies of gene expression in colon cancer, but few studies involved multiple gene expression files and focused on an early diagnosis of the disease. Hence, we performed this study in order to deepen the understanding of the underlying mechanism and provide novel biomarkers for early diagnosis and prognosis of the disease.

RETRACTED

## 2. Materials and Methods

### 2.1. Microarray Data

We first searched the GEO database [15] and identified three microarray datasets (GSE110224, GSE44076, and GSE47063) [16–18] describing gene expression differences between COAD and normal colon tissue. GSE110224 is based on platform GPL570 ([HG-U133_Plus_2] Affymetrix Human Genome U133 Plus 2.0 Array), GSE44076 is based on platform GPL13667 ([HG-U219] Affymetrix Human Genome U219 Array), and GSE47063 is based on platform GPL6102 (Illumina human-6 v2.0 expression beadchip). All data are freely available online.

### 2.2. DEG Identification

GEO2R is commonly used to process sample information from GEO series and to identify DEGs among user-defined groups. After screening the sample information in the three data sets, only the COAD samples and the corresponding normal tissues were included. After GEO2R analysis, DEGs were obtained by intersecting genes with an adjusted *P* < 0.05 and |logFC| ≥ 1 in each data set using a Venn diagram.

### 2.3. Gene Ontology and Pathway Enrichment Analysis of DEGs

Metascape [19] is an open access online tool for comprehensive gene list annotation and analysis. In this study, DEG pathway and process enrichment analyses were performed using Metascape. The parameters were set as follows: 3 for min overlap, 1.5 for min enrichment, and *P* value cutoff of 0.05. The enrichment results were presented as bar charts. Corresponding network graph nodes with similarity degree more than 0.3 were connected with curved edges. Edge thickness was positively correlated with the degree of similarity.

### 2.4. PPI Network Construction and Module Analysis

The Search Tool for the Retrieval of Interacting Genes (STRING) database [20] was used to construct the PPI network with an interaction score > 0.4. Then, Cytoscape (Version 3.7.2) [21] software was used to visualise and analyse PPI networks. Molecular Complex Detection (MCODE) (Version 1.6) [22], a Cytoscape plugin, was used to identify the most significant gene module in colon cancer. Then, we annotated the function of the module genes using Metascape.

### 2.5. Hub Gene Selection and Analysis

CytoHubba (Version 0.1) [23], a Cytoscape plugin, was used to identify the network hub genes. We used a degree-ranked method to identify hub genes with a criterion of degree no less than 67. ClueGO [24] is another Cytoscape plugin that can creates and visualises functionally grouped networks of biological terms and pathways. The CluePedia [25] Cytoscape plugin is a functional extension of ClueGO and a search tool for new markers potentially associated with pathways. In our study, ClueGO (Version 2.5.6) and CluePedia (Version 1.5.6) were used to analyse the biological processes and pathway enrichment of hub genes.

RETRACTED

### 2.6. Analysis of Prognostic Value of Hub Genes

GEPIA [26] is an integrated bioinformatics analysis tool which was designed for transforming genomic big data into intuitive graphics. In this study, GEPIA was used to perform survival analysis based on gene expression. *P* < 0.05 was considered statistically significant.

### 2.7. Hub Gene Expression Analysis and ROC Curve Analysis

UALCAN [27] is a comprehensive interactive online resource which contains clinical data from 31 cancer types from the TCGA database. We used UALCAN to perform differential expression analysis of the hub genes and their association with clinicopathological parameters of COAD patients. Moreover, the Human Protein Atlas [28] is a website for users to freely access data for exploration of the human proteome, which contains transcriptome data from 17 main cancer types using data from nearly 8000 patients. In this study, histopathological data of the hub genes were downloaded and used for direct comparison the protein expression. We selected an additional dataset for ROC curve analysis of diagnostic accuracy for the hub genes. GSE87211 [29] is based on platform GPL13497 (Agilent-026652 Whole Human Genome Microarray 4x44K v2). All data are freely available online.

### 2.8. Analysis of Alterations of Hub Genes

cBioPortal [30] is a free web server for interactively exploring cancer genomics datasets. In this study, cBioPortal was utilised to predict the genetic alterations of eight hub genes in 378 COAD samples (TCGA, PanCancer Atlas) which contained mutations and putative copy-number alterations from GISTIC and mRNA expression *z*-scores (RNASeq V2 RSEM) with a *z*-score threshold ±2.0.

### 2.9. Statistical Analysis

Microarray data analysis was performed by using GEO2R. GEOquery R package was used to transform the original data into R data structure, and then, the statistical test of limma (linear models for microarray analysis) R package was used to identify DEGs. Survival analysis was performed by using GEPIA and log-rank test. The transcripts per million (TPM) expression value and *t*-test were used for analysis of the relationship between hub genes expression and clinicopathological parameters. SPSS 26.0 was used for ROC curve analysis. *P* < 0.05 was considered statistically significant.

## 3. Results

### 3.1. DEGs in Colon Cancer

Among the three datasets (GSE110224, GSE44076, and GSE47063), there were 127 COAD tissues and 117 normal tissues. After GEO2R analysis, we screened 1617 DEGs (745 upregulated and 872 downregulated) from GSE110224, 4450 DEGs (2095 upregulated and 2355 downregulated) from GSE44076, and 2259 DEGs (1056 upregulated and 1203 downregulated) from GSE47063. Then, 436 DEGs were obtained by overlapping the three dataset results, including 267 downregulated genes (Figure 1(a)) and 169 upregulated genes (Figure 1(b)).

RETRACTED

### 3.2. DEG Gene Ontology (GO) and Pathway Enrichment in Colon Cancer

The top 20 GO items were divided into 3 categories: biological processes (14 items), cellular components (4 items), and molecular functions (2 items; Table 1 and Figures 2(a) and 2(b)). The DEGs were mainly enriched in cell cycle, transcriptional regulation, and ion transport. Enriched biological processes included cell cycle phase transition, nuclear division, meiotic nuclear division, cytokinesis, DNA replication, negative regulation of cell proliferation, regulation of reproductive process, regulation of MAPK cascade, positive regulation of transferase activity, bicarbonate transport, inorganic ion homeostasis, cellular response to organic cyclic compound, cellular response to nitrogen compound, and mesenchymal cell differentiation. Cellular component analysis showed that the DEGs were significantly enriched in the apical part of the cell, spindle, microvillus, and basolateral plasma membrane. Molecular functions of these genes were histone kinase activity and activity of hydrolase acting on ester bond.

The top 20 Kyoto Encyclopedia of Genes and Genomes (KEGG) and Reactome pathways were shown in Table 2 and Figures 2(c) and 2(d). DEGs were mainly enriched for terms associated with the cell cycle, reversible hydration of carbon dioxide, proximal tubule bicarbonate reclamation, transport of small molecules, cyclin A/B1/B2 associated events during G2/M transition, and regulation of TP53 activity through phosphorylation pathway.

### 3.3. DEG PPI Network and Modules

A PPI network composed of 369 nodes and 2708 edges was constructed (Figure 3). Then, MCODE was used to isolate the significant network modules. We selected the most significant module with the highest degree (Figure 4(a)) and functionally annotated the involved genes (Table 3). GO enrichment analysis showed that the genes were mainly enriched in biological processes, including chromosome segregation, cell cycle phase transition, positive regulation of cell cycle, DNA replication, meiotic cell cycle, attachment of spindle microtubules to kinetochore, DNA conformation change, signal transduction by p53 class mediator, positive regulation of transferase activity, sister chromatid cohesion, cytokinetic process, and protein localisation to cytoskeleton. Cellular component analysis showed that these genes were mainly enriched in the spindle, midbody, kinesin complex, and intercellular bridge. Molecular function analysis showed that these genes were mainly enriched in catalytic activity, acting on DNA, and chromatin binding. Pathway analysis revealed that these genes were mainly enriched in cyclin A/B1/B2-associated events during G2/M transition and APC-Cdc20-mediated degradation of Nek2A.

RETRACTED

### 3.4. Hub Genes

According to the node degree calculated by CytoHubba, 20 hub genes were screened out, and they were all upregulated (Figure 4(b)). The gene symbols and corresponding degree were shown in Table 4. Functional annotation of the 20 hub genes was shown in Figures 4(c) and 4(d). Heat map visualisation showed that the expression of these 20 hub genes in COAD tissues was higher than in normal tissues (Figure 4(e)).

### 3.5. Survival Based on Hub Gene Expression

Because several hub genes were closely related to the cell cycle, we further analysed their survival curves using the GEPIA database. Our results showed that overexpression of six hub genes influenced COAD prognosis, including *CCNB1*, *CCNA2*, *AURKA*, *NCAPG*, *DLGAP5*, and *CENPE*. Overexpression of the six genes was associated with favourable overall survival (OS) of colon cancer patients (Figures 5(a)–5(f)). Additionally, *AURKA* and *CENPE* overexpressions showed a favourable prognosis of disease-free survival (DFS) in COAD patients (Figures 5(g) and 5(h)).

### 3.6. Differential Expression of Hub Genes

UALCAN was used to analyse mRNA expression of the identified hub genes. We found 5 hub genes were related to clinicopathological parameters, including *CDK1*, *CCNB1*, *CCNA2*, *MAD2L1*, and *DLGAP5*. Additionally, we observed that these five genes were significantly overexpressed in tumour tissues (Figures 6(a), 6(d), 6(g), 6(j), and 6(m)). Then, we analysed their mRNA expression under different clinicopathological parameters. Our results revealed that the mRNA expression of the five genes was significantly correlated with the clinical stage, and that the highest mRNA expression appeared in the first tumour stage (Figures 6(b), 6(e), 6(h), 6(k), and 6(n)). Moreover, the mRNA expression of the five genes showed a significant correlation with lymph node metastasis, and the highest mRNA expression appeared at the N0 phase (Figures 6(c), 6(f), 6(i), 6(l), and 6(o)).

Moreover, we analysed the protein expressions of hub genes using histopathological images from HPA. Our results showed that CDK1 staining was low in normal tissues and moderate in COAD tissues (Figure 7(a)). CCNB1 and CCNA2 staining were moderate in normal colon tissues, whereas high staining was observed in COAD tissues (Figures 7(b) and 7(c)). DLGAP5 staining was not detected in normal tissues, while moderate staining was observed in COAD tissues (Figure 7(d)). MAD2L1 was moderately stained in both tumour and normal tissues (Figure 7(e)).

RETRACTED

In order to further test the diagnostic efficacy of these hub genes for colon cancer, ROC curve analysis was performed on these five genes (Figure 8). We used gene expression data from GSE87211 for analysis. The dataset contained 363 cases (203 colon tumours and 160 healthy mucosa). AUCs were used to assess the diagnostic accuracy. ROC analysis showed that AUCs for *CDK1*, *CCNB1*, *CCNA2*, *MAD2L1*, and *DLGAP5* were 0.928 (95% CI: 0.901-0.956), 0.931 (95% CI: 0.905-0.956), 0.904 (95% CI: 0.847-0.934), 0.917 (95% CI: 0.887-0.947), and 0.911 (95% CI: 0.881-0.940), respectively.

### 3.7. Alteration of Hub Genes

We also analysed alterations of the six prognostic hub genes *CCNB1*, *CCNA2*, *AURKA*, *NCAPG*, *DLGAP5*, and *CENPE* together with the five hub genes which were associated with clinicopathological parameters: *CDK1*, *CCNB1*, *CCNA2*, *MAD2L1*, and *DLGAP5*. Eight hub genes including *CDK1*, *CCNB1*, *CCNA2*, *AURKA*, *MAD2L1*, *NCAPG*, *DLGAP5*, and *CENPE* were detected by cBioPortal.

Altogether, 378 samples of COAD were included, and our analysis revealed that the hub genes were altered in 42.86% of the 378 samples. *AURKA* (28%) was the most frequently altered gene of the eight hub genes (Figure 9).

## 4. Discussion

Colon cancer was the fourth most commonly diagnosed malignant tumour worldwide in 2018, with increasing incidence in countries undergoing major developmental transition [31]. Due to a lack of specific symptoms for early detection, patients are usually diagnosed at an advanced stage which leads to a poor prognosis [32]. Therefore, it is crucial to uncover the underlying molecular mechanism and to explore key biomarkers for early colon cancer diagnosis.

In this study, we analysed three microarray datasets that included 127 tumours and 117 normal samples. A total of 436 DEGs were screened. Functional annotation showed that the DEGs were mainly enriched in biological processes associated with cell cycle phase transition, nuclear division, positive regulation of transferase activity, meiotic nuclear division, and DNA replication. These results suggested that these genes were closely related to the cell cycle. Many studies indicated that dysregulation of cell cycle progression was closely related to cancer progression [33, 34]. Finetti et al. [35] found that several genes participated in regulating the cell cycle, like *CDK1* and *AURKA*. Moreover, their expressions were correlated with breast cancer prognosis. In our colon cancer study, we obtained many DEGs involved in cell cycle progression, including *CCND1*, *BLM*, *BUB1*, *BUB1B*, *CCNA2*, *CCNB1*, *CDK1*, and *CDC20*. Some genes were closely related to the transformation of cancer. For example, *CCND1* belonged to the cyclin family whose members were characterised by dramatic periodicity in protein abundance throughout the cell cycle. Deregulation of *CCND1* was observed frequently in numerous human cancers, including pancreatic cancer, head and neck squamous cell carcinoma, breast cancer, and colorectal carcinoma [36, 37]. Accumulation of *CCND1* in the nucleus caused uncontrolled cell cycle progression and acted as a tumour-initiating event [38]. Overexpression of cyclin D1 (T286A), an oncogenic mutant allele of *CCND1*, promoted stabilization and overexpression of the DNA replication licensing factor, Cdt1, by inhibiting its proteolysis. This caused DNA rereplication and damage and resulted in cellular aneuploidy, genomic instability, and further neoplastic growth [39]. Cyclin dependent kinases (CDKs) were necessary functional partner kinases with cyclin D1. Thus, CDK inhibitors would be an effective drug for targeting malignant tumours [40]. However, given the development of resistance and side effects of CDK inhibitors, further research is warranted [36].

RETRACTED

Pathway analysis also revealed that DEGs were mainly enriched for terms associated with the cell cycle pathway. Cyclin A/B1/B2-associated events in the “G2/M transition” and “Regulation of TP53 Activity through Phosphorylation” pathways were closely related to tumourigenesis. Like the cyclin D1 mentioned above, cyclins A/B1/B2 were also cyclin members that binded to CDKs and regulated the cell cycle. Abundant evidence showed that G2/M phase arrest was closely related to the inhibition of tumour cell proliferation [41, 42]. Additional studies focusing on cyclins are aimed at identifying novel therapeutic strategies for cancer treatment. Ma [43] revealed that the microRNA miR-219-5p downregulated *CCNA2* expression and induced G2/M phase arrest to inhibit tumour formation in oesophageal cancer. Tu et al. [44] found *CCNA2* was downregulated by the small molecule FH535 in colorectal cancer, which caused G2/M phase arrest and inhibited tumour proliferation. Thus, inhibiting *CCNA2* and *CCNB1* may contribute to the development of novel anticancer drugs. The p53 signalling pathway significantly contributed to cell cycle regulation, suppression of tumour expression, metabolism, aging, development, and reproduction [45]. Phosphorylation of p53 protein stabilized the protein and extended its half-life, thus, causing cell cycle arrest, apoptosis, and inhibited tumour cell proliferation [46]. A study of natural polyphenols as anticancer agents revealed that polyphenols could induce apoptosis, which was achieved by stabilizing p53 protein through phosphorylation and showed remarkable effects in human gastric carcinoma cells [47]. We also identified some pathways associated with metabolism, including triglyceride metabolism, carnitine metabolism, regulation of lipolysis in adipocytes, and phase I—functionalization of compounds. Among these pathways, we found that *FABP4*, which encoded fatty acid binding protein, was involved in fatty acid uptake, transport, and metabolism and was related to tumour metastasis. Gharpure et al. [48] observed that overexpression of *FABP4* played a key role in aggressive metastasis of ovarian cancer via various metabolites and protein pathways. Likewise, *FABP4* had crucial effects on adipocyte-induced cholangiocarcinoma metastasis [49]. Collectively, metabolic disorder was among the leading causes of tumour development. Thus, the study of tumour metabolism may provide new targets for tumour treatment.

RETRACTED

The PPI network was built using STRING. Twenty hub genes were screened, and their functional annotations were most closely related to the cell cycle. Survival analysis showed that higher mRNA expression of six hub genes was significantly related to longer OS in colon cancer patients, including *CCNB1*, *CCNA2*, *AURKA*, *NCAPG*, *DLGAP5*, and *CENPE*. Moreover, *AURKA* and *CENPE* exhibited favourable effects on both OS and DFS. Studies showed that *CCNB1* was highly expressed in colorectal cancer tissues and was negatively correlated with tumour invasion and distant metastasis, which may be caused by regulating the expression of E-cadherin [50]. This was consistent with our findings. A murine colorectal cancer model showed that *CCNA2* deletion in colonic epithelial cells promoted the development of dysplasia and adenocarcinomas [51]. Analysis of *CCNA2* expression in clinical samples revealed that higher expression of *CCNA2* in tumours of stage 1 or 2 colon cancer patients is compared with stage 3 or 4 patients [51], which was also consistent with our results. However, previous studies had shown that *CCNA2* was tumour-promoting and associated with advanced tumour stage and tumour development [52, 53]. This was inconsistent with our results, which may be due to the heterogeneity of the sample. Besides, high expression of *DLGAP5* was associated with poor prognosis in well differentiated colon cancer, whereas the prognosis was better in some molecular subtypes of colon cancer, such as patients with a stem cell gene signature [54] and Budinska subtypes A (surface crypt-like) [55]. In our study, *AURKA* exhibited favourable prognostic effects. Interestingly, *AURKA* was upregulated across cancer types, but was only positively associated with prognosis in colon cancer patients [56]. Current studies supported that *AURKA* was associated with the development of colorectal cancer by causing genomic instability [57], but high expression of *AURKA* in colon cancer enhanced the chemotherapy sensitivity of platinum drugs by inhibiting the expression of TP53-regulated DNA damage response genes, which may explain the corresponding better prognosis [56]. However, it has also been reported that high expression of *AURKA* is associated with poor prognosis in colon cancer patients with liver metastasis [58]. Therefore, there was still controversy, and further exploration was needed. *NCAPG and CENPE* have also been reported to play a role in various types of cancer [59, 60], but the underlying mechanisms behind the observed changes in prognosis remain unknown. In summary, these 6 hub genes were significantly associated with the prognosis of colon cancer and may serve as potential prognostic markers as well as therapeutic targets, but further studies were needed to explain and verify their underlying mechanisms.

RETRACTED

For early COAD diagnosis, we identified *CDK1*, *CCNB1*, *CCNA2*, *MAD2L1*, and *DLGAP5*, which were closely related to clinicopathological parameters. *CDK1* plays a key role in the regulation of eukaryotic cell cycle and is essential for G1/S and G2/M transition of eukaryotic cell cycle [61]. Many biological experiments have demonstrated that *CDK1* is highly expressed in colon cancer cells [62, 63] and participates in apoptosis. *CDK1* may act as a potential diagnostic and therapeutic target in view of its extensive involvement in the regulation of colorectal cancer development and progression [62]. *CCNB1* and *CCNA2* are closely related to mitosis. In addition to colon cancer, they have also been found to be highly expressed in pancreatic cancer [64], breast cancer [65], lung cancer [66], and many other cancers, suggesting their potential diagnostic value. *MAD2L1* was highly expressed in active proliferating colon cancer cells, and its expression level gradually increased with the stage of colon cancer [67]. *DLGAP5* was involved in cell proliferation (ClueGO analysis: mitotic chromosome movement towards spindle pole) which was highly expressed in colon cancer cells [54, 68]. One study showed that *DLGAP5* was overexpressed in 293 T cells, resulting in excessive cell proliferation, which may play a potential role in carcinogenesis [69]. In summary, our results showed that both the mRNA and protein expressions of these five hub genes were higher in tumour tissue than in normal tissue, which indicated that the hub genes may be closely related to COAD progression and the possibility of five gene biomarkers in the diagnosis of CRC. Previous studies observed that the expression of these genes was correlated with tumour size and stage [52, 54, 70]. In our study, we found that mRNA expression of the five hub genes was significantly related to mild clinical pathological parameters, so these genes may play an important role in the early diagnosis of colon cancer. In addition, AUCs of these five genes were all greater than 0.9 in ROC curve analysis, which further verified the favourable diagnostic accuracy of these five genes. The relationship between these genes and COAD has not yet been fully determined, but our data indicate that the increased expression in early COAD stages may provide an indicator for early diagnosis. At present, machine learning and deep learning are widely used in disease diagnosis [71, 72]. Deep learning, with its ability to process large-scale data, is a powerful solution for tissue classification and segmentation of histopathological images of colon cancer and other diseases [73, 74].

RETRACTED

We finally performed alteration analysis of eight hub genes which showed significant effects on survival analysis, including *CDK1*, *CCNB1*, *CCNA2*, *AURKA*, *MAD2L1*, *NCAPG*, *DLGAP5*, and *CENPE*. The result showed that more than 40% of the patient tumours analysed had at least one hub gene alteration. *AURKA* was the most frequently altered (28%) of the 8 hub genes. The protein encoded by this gene is a cell cycle-regulated kinase that appears to be involved in spindle assembly, cytokinesis, centrosome maturation, and separation [75]. In our study, *AURKA* exhibited favourable effects on both OS and DFS. Previous studies showed that *AURKA* was frequently upregulated and correlated with prognosis in several types of cancers, which may reveal an important role in human cancer [76, 77].

There were some limitations in this study. First, all the data analysed in our study was retrieved from online databases. Thus, further studies with larger sample sizes and biological experiments were required to validate our findings. Our future research will focus on experimental verification of these results. Second, we did not explore the underlying mechanisms of hub genes in COAD. Future studies should investigate the detailed mechanism between hub genes and COAD.

In conclusion, our study identified and analysed DEGs and 20 core genes associated with COAD, which might deepen the understanding of carcinogenesis and provide indicators for prognosis and early diagnosis of the disease.

RETRACTED

## Figures and Tables

**Figure 1:** Venn diagram of DEGs from three datasets. (a) 267 downregulated DEGs. (b) 169 upregulated DEGs. Abbreviations: DEGs: differentially expressed genes.

**Figure 2:** DEG and neighbouring gene enrichment analysis in COAD using Metascape. (a) Heatmap of GO enriched terms coloured by *P* value. (b) Network of GO enriched terms coloured by *P* value. Each node represents an enriched term. Dark colours indicate increased statistical significance. (c) Heatmap of KEGG and Reactome enriched terms coloured by *P* value. (d) Network of KEGG and Reactome enriched terms coloured by *P* value. Each node represents an enriched term. Darker colour indicates more statistical significance. Abbreviations: DEGs: differentially expressed genes; COAD: colon adenocarcinoma; GO: Gene Ontology; KEGG: Kyoto Encyclopedia of Genes and Genomes.

**Figure 3:** PPI network of DEGs, containing 369 nodes and 2708 edges. Red represents upregulated genes. Blue represents downregulated genes. Abbreviations: PPI: protein-protein interaction; DEGs: differentially expressed genes.

**Figure 4:** The most significant module gene network and hub genes analysis. (a) The most significant module in the PPI network contains 62 nodes and 1708 edges. (b) Network of 20 hub genes. Darker colours represent higher scores. (c) Biological process annotation of hub genes using ClueGO and CluePedia. *P* < 0.01 was considered statistically significant. (d) KEGG annotation of hub genes using ClueGO and CluePedia. *P* < 0.01 was considered statistically significant. (e) Heatmap of the top 20 hub genes was constructed using the UALCAN database. Abbreviations: PPI: protein-protein interaction; KEGG: Kyoto Encyclopedia of Genes and Genomes.

**Figure 5:** Overall survival of the hub genes in COAD patients. (a)–(f) *CCNB1*, *CCNA2*, *AURKA*, *NCAPG*, *DLGAP5*, and *CENPE* showed a significant difference in overall survival (OS). High expression of the 6 genes indicated favourable OS in COAD (*P* < 0.05). (g, h) *AURKA* and *CENPE* showed statistically significant association with disease-free survival (DFS) and indicated favourable disease-free survival in COAD (*P* < 0.05). Abbreviations: COAD: colon adenocarcinoma.

**Figure 6:** Differential expression analysis of the 5 hub genes was performed by UALCAN. (a, d, g, j, and m) mRNA expression of the five genes was overexpressed in colon cancer compared to normal colon tissues. (b, e, h, k, and n) mRNA expression of the five genes was significantly related to individual cancer stage, with the highest expressions tending to appear at stage 1. (c, f, i, l, and o) mRNA expression of the five genes was significantly related to nodal metastasis status, and the highest mRNA expression tended to appear at the N0 phase. ^∗^*p* < 0.05, ^∗∗^*p* < 0.01, ^∗∗∗^*p* < 0.001.

RETRACTED

**Figure 7:** Protein expression analysis of the 5 hub genes was performed using the HPA database. Except for MAD2L1, the other 4 proteins showed a higher degree of staining in tumour tissue compared to normal tissues.

**Figure 8:** ROC curves analysis of the five hub genes, *CDK1*, *CCNB1*, *CCNA2*, *MAD2L1*, and *DLGAP5*. AUCs were used to assess the five hub genes, and the results showed high diagnostic accuracy.

**Figure 9:** Alterations of the eight hub genes analysed by cBioPortal. (a) OncoPrint of genetic alterations in 378 COAD cases. (b) Alteration frequency of eight hub genes. Gene expression was altered in 42.86% of 378 cases. Abbreviations: COAD: colon adenocarcinoma.

**Table 1:** Gene ontology (GO) annotation of DEGs in COAD.

GO	Category	Description	Count	%	Log10(*P*)	Log10(*q*)
GO:0044770	GO biological processes	Cell cycle phase transition	45	10.32	-14.12	-10.06
GO:0000280	GO biological processes	Nuclear division	36	8.26	-14.06	-10.06
GO:0051347	GO biological processes	Positive regulation of transferase activity	37	8.49	-8.32	-5.38
GO:0140013	GO biological processes	Meiotic nuclear division	17	3.90	-7.60	-4.94
GO:0006260	GO biological processes	DNA replication	19	4.36	-6.27	-3.79
GO:2000241	GO biological processes	Regulation of reproductive process	14	3.21	-6.22	-3.75
GO:0015701	GO biological processes	Bicarbonate transport	8	1.83	-6.06	-3.60
GO:0008285	GO biological processes	Negative regulation of cell proliferation	34	7.80	-5.72	-3.29
GO:0048762	GO biological processes	Mesenchymal cell differentiation	16	3.67	-5.61	-3.19
GO:0071407	GO biological processes	Cellular response to organic cyclic compound	27	6.19	-5.60	-3.19
GO:0043408	GO biological processes	Regulation of MAPK cascade	33	7.57	-5.52	-3.13
GO:0098771	GO biological processes	Inorganic ion homeostasis	33	7.57	-5.46	-3.08
GO:1901699	GO biological processes	Cellular response to nitrogen compound	30	6.88	-5.39	-3.02
GO:0000910	GO biological processes	Cytokinesis	14	3.21	-5.33	-2.97
GO:0045177	GO cellular components	Apical part of cell	34	7.80	-12.92	-9.27
GO:0005819	GO cellular components	Spindle	27	6.19	-9.32	-6.23
GO:0005902	GO cellular components	Microvillus	13	2.98	-8.20	-5.35
GO:0016323	GO cellular components	Basolateral plasma membrane	16	3.67	-5.41	-3.04
GO:0035173	GO molecular functions	Histone kinase activity	6	1.38	-6.46	-3.97
GO:0016788	GO molecular functions	Hydrolase activity, acting on ester bonds	33	7.57	-5.61	-3.19

Abbreviations: DEGs: differentially expressed genes; COAD: colon adenocarcinoma.

**Table 2:** KEGG and Reactome annotation of DEGs in COAD.

GO	Category	Description	Count	%	Log10(*P*)	Log10(*q*)
hsa04110	KEGG pathway	Cell cycle	16	3.67	-9.05	-6.08
hsa04964	KEGG pathway	Proximal tubule bicarbonate reclamation	5	1.15	-4.32	-2.26
hsa04923	KEGG pathway	Regulation of lipolysis in adipocytes	6	1.38	-3.38	-1.5
hsa04960	KEGG pathway	Aldosterone-regulated sodium reabsorption	5	1.15	-3.3	-1.48
hsa04978	KEGG pathway	Mineral absorption	5	1.15	-2.65	-1.03
R-HSA-1640170	Reactome gene sets	Cell cycle	41	9.4	-10.9	-7.44
R-HSA-1475029	Reactome gene sets	Reversible hydration of carbon dioxide	5	1.15	-5.87	-3.47
R-HSA-382551	Reactome gene sets	Transport of small molecules	29	6.65	-4.18	-2.14
R-HSA-69273	Reactome gene sets	Cyclin A/B1/B2 associated events during G2/M transition	5	1.15	-4.13	-2.11
R-HSA-6804756	Reactome gene sets	Regulation of TP53 activity through phosphorylation	8	1.83	-3.58	-1.64
R-HSA-109582	Reactome gene sets	Haemostasis	24	5.5	-3.35	-1.5
R-HSA-8979227	Reactome gene sets	Triglyceride metabolism	5	1.15	-3.3	-1.48
R-HSA-418594	Reactome gene sets	G alpha (i) signalling events	17	3.9	-2.89	-1.16
R-HSA-420029	Reactome gene sets	Tight junction interactions	4	0.92	-2.76	-1.09
R-HSA-200425	Reactome gene sets	Carnitine metabolism	3	0.69	-2.74	-1.09
R-HSA-420092	Reactome gene sets	Glucagon-type ligand receptors	4	0.92	-2.55	-0.95
R-HSA-211945	Reactome gene sets	Phase I—functionalization of compounds	7	1.61	-2.5	-0.91
R-HSA-6785807	Reactome gene sets	Interleukin-4 and interleukin-13 signalling	7	1.61	-2.46	-0.88
R-HSA-983189	Reactome gene sets	Kinesins	5	1.15	-2.38	-0.82
R-HSA-422085	Reactome gene sets	Synthesis, secretion, and deacylation of ghrelin	3	0.69	-2.34	-0.8

Abbreviations: KEGG: Kyoto Encyclopedia of Genes and Genomes; DEGs: differentially expressed genes; COAD: colon adenocarcinoma.

RETRACTED

**Table 3:** Functional annotation of the genes involved in the most significant module.

GO	Category	Description	Count	%	Log10(*P*)	Log10(*q*)
GO:0007059	GO biological processes	Chromosome segregation	29	46.77	-37.06	-32.66
GO:0044770	GO biological processes	Cell cycle phase transition	33	53.23	-35.09	-31.16
GO:0045787	GO biological processes	Positive regulation of cell cycle	17	27.42	-15.9	-13.21
GO:0006260	GO biological processes	DNA replication	14	22.58	-14.21	-11.7
GO:0051321	GO biological processes	Meiotic cell cycle	12	19.35	-11.78	-9.35
GO:0008608	GO biological processes	Attachment of spindle microtubules to kinetochore	7	11.29	-11.68	-9.27
GO:0071103	GO biological processes	DNA conformation change	12	19.35	-10.45	-8.08
GO:0072331	GO biological processes	Signal transduction by p53 class mediator	10	16.13	-8.81	-6.51
GO:0051347	GO biological processes	Positive regulation of transferase activity	14	22.58	-8.75	-6.45
GO:0007062	GO biological processes	Sister chromatid cohesion	6	9.68	-7.87	-5.62
GO:0032506	GO biological processes	Cytokinetic process	5	8.06	-7.29	-5.1
GO:0044380	GO biological processes	Protein localisation to cytoskeleton	5	8.06	-6.41	-4.27
GO:0005819	GO cellular components	Spindle	23	37.1	-25.83	-22.66
GO:0030496	GO cellular components	Midbody	14	22.58	-16.65	-13.9
GO:0005871	GO cellular components	Kinesin complex	5	8.06	-6.53	-4.38
GO:0045171	GO cellular components	Intercellular bridge	5	8.06	-5.97	-3.86
GO:0140097	GO molecular functions	Catalytic activity, acting on DNA	7	11.29	-5.87	-3.78
GO:0003682	GO molecular functions	Chromatin binding	10	16.13	-5.86	-3.76
R-HSA-69273	Reactome gene sets	Cyclin A/B1/B2 associated events during G2/M transition	4	6.45	-6.32	-4.18
R-HSA-179409	Reactome gene sets	APC-Cdc20 mediated degradation of Nek2A	4	6.45	-6.32	-4.18

Abbreviations: GO: Gene Ontology.

**Table 4:** Top 20 hub genes and corresponding degree.

Gene symbol	Gene description	Score
CDK1	Cyclin dependent kinase 1	78
CCNB1	Cyclin B1	76
CCNA2	Cyclin A2	75
AURKA	Aurora kinase A	75
CDC20	Cell division cycle 20	74
AURKB	Aurora kinase B	72
TPX2	TPX2 microtubule nucleation factor	71
BUB1	BUB1 mitotic checkpoint serine/threonine kinase	70
CDC45	Cell division cycle 45	70
MAD2L1	Mitotic arrest deficient 2 like 1	69
KIF2C	Kinesin family member 2C	69
NCAPG	Non-SMC condensin I complex subunit G	69
DLGAP5	DLG associated protein 5	69
FOXM1	Forkhead box M1	69
CENPF	Centromere protein F	68
CENPE	Centromere protein E	68
BUB1B	BUB1 mitotic checkpoint serine/threonine kinase B	68
TTK	TTK protein kinase	68
ASPM	Abnormal spindle microtubule assembly	68
KIF20A	Kinesin family member 20A	67

## Data Availability

All The data used to support the findings of this study are available online.
